# Plumbagin relieves rheumatoid arthritis through nuclear factor kappa-B (NF-κB) pathway

This article has been retracted.

**DOI:** 10.1080/21655979.2022.2081756

**Published:** 2022-06-02

**Authors:** Chang Shu, Jun Chen, Meiyan Lv, Yiyuan Xi, Jujia Zheng, Xiangwei Xu

**Affiliations:** a Department of Orthopaedic, The First People’s Hospital of Yongkang, Yongkang, Zhejiang, China; b Department of Pharmacy, The First People’s Hospital of Yongkang, Yongkang, Zhejiang, China; c Department of Clinical Laboratory, The First People’s Hospital of Yongkang, Yongkang, Zhejiang, China; d School of Pharmaceutical Sciences, Wenzhou Medical University, Wenzhou, Zhejiang, China

**Keywords:** Rheumatoid arthritis, plumbagin, inflammation, NF-κB

## Abstract

This study aimed to explore the effects of plumbagin on rheumatoid arthritis (RA) and its mechanism. The RA cell model was simulated following the treatment of interleukin-1β (IL-1β). After the treatment of various concentrations of plumbagin, the impact of plumbagin on the cell viability was examined by 3-(4,5-Dimethylthiazol-2-yl)-2,5-diphenyltetrazolium bromide (MTT) assay. The collagen-induced arthritis (CIA) model was established using the solution of bovine type II collagen. Hematoxylin-eosin staining was used to observe the changes of ankle joint tissue, while enzyme-linked immunosorbent assay and western blot were applied to detect the level of inflammatory cytokines. Plumbagin inhibited the viability of human fibroblast-like synoviocytes (HFLS) at the concentration of 1 ~ 3.5 μM. The inhibitory effect of 1 μM plumbagin on cell proliferation was similar to that of methotrexate, the drug used as the positive control. Plumbagin downregulated the levels of inflammatory cytokines and matrix metalloproteinases (MMPs) in IL-1β-treated HFLS, and suppressed the activation of IκB and nuclear factor kappa-B (NF-κB) as well as the entry of p65 into the nucleus. It was also demonstrated in animal experiments that plumbagin inhibited the activation of NF-κB pathway, down-regulated the levels of tumor necrosis factor-α (TNF-α), interleukin-6 (IL-6) and MMPs, and alleviated joint damage in CIA-modeled mice. Collectively speaking, plumbagin might down-regulate the levels of inflammatory cytokines and MMPs through inhibiting the activation of the NF-κB pathway, thereby attenuating RA-induced damage to cells and joints.

**Abbreviations**: CIA: Collagen-induced arthritis; ELISA: Enzyme-linked immuno sorbent assay; HFLS: Human fibroblast-like synoviocytes; IL-6: Interleukin-6; IL-1β: Interleukin-1β; NF-κB: nuclear factor kappa-B; MTT: 3-(4,5-Dimethylthiazol-2-yl)-2,5-diphenyltetrazolium bromide; MMPs: Matrix metalloproteinase; OD: Optical density; RA: Rheumatoid arthritis; SDS: Sodium dodecyl sulfate; SD: Standard deviation; TNF-α: Tumor necrosis factor-α; PVDF: Polyvinylidene fluoride.

## Highlights

- Plumbagin inhibits the growth of RA-modeled HFLS.
- Plumbagin attenuates inflammatory and MMPs levels in IL-1β-induced RA-modeled HFLS.
- Plumbagin diminishes the levels of inflammatory factors and MMPs of CIA mice.
- Plumbagin alleviates rheumatoid arthritis in CIA mice via regulating NF-κB pathway.

## Introduction

Rheumatoid arthritis (RA) is a heterogeneous, systemic autoimmune disease characterized by symmetrical joint swelling and pain [1]. In the advanced stage of RA, joint rigidity or deformity may occur, which causes the severely impaired joint function and high morbidity [2]. As a systemic disease, RA also induces the development of other tissue diseases, such as cardiovascular disease and interstitial lung disease [3,4].

Although previous research has suggested that gene, infection, hormone levels, environmental factors, malnutrition, and trauma can induce RA [5,6], the etiology of RA remains dim and awaits to be elucidated. The typical characteristics of RA refers to synovial inflammation, synovial hyperplasia, cartilage absorption, and bone destruction [1,5,6]. Meanwhile, it has been proposed that some cytokines secreted by the macrophages and chondrocytes, including tumor necrosis factor-α (TNF-α), interleukin-1β (IL-1β), interleukin-6 (IL-6), and matrix metalloproteinase (MMPs), are closely related to RA [7,8].

Plumbagin (5-hydroxy-2-methyl-1,4-naphthoquinone) is a plant-derived quinoid component from the genera of *Drosera* and *Plumbago zeylanica*, which possesses various biological activities such as anti-tumor and anti-inflammation, with an alleviative effect on the oxidative stress [9,10]. A recent study indicated that plumbagin could notably reduce the secretion of MMP-1, MMP-3, MMP-13 as well as the inflammatory response of IL-1β-induced chondrocytes, and greatly alleviate the symptoms of mice with osteoarthritis [11]. Plumbagin also inhibits the secretion of IL-1 and IL-6 in microglial cells following the induction of lipopolysaccharide [12]. Guo et al [13]additionally put forward that plumbagin can suppress the levels of TNF-α and IL-6 by activating nuclear factor (erythroid-derived 2)-like 2 (Nrf-2), and alleviate oxidative stress and inflammation of H_2_O_2_-stimulated chondrocytes. In accordance with these studies, we hypothesized that plumbagin might exert an anti-inflammatory effect on RA.

On the basis of above, the effects and possible mechanism of plumbagin on fibroblast-like synoviocytes and RA-modeled mice were investigated and analyzed in this paper so as to provide the theoretical basis and a possibly viable method for the treatment of RA in clinic.

## Methods and materials

### Cell culture and experiment design

RA human fibroblast-like synoviocytes (HFLS-RAs) (ATCC, USA) were cultured in RPMI-1640 (Thermo Fisher, Waltham, Massachusetts, USA) containing 2% fetal bovine serum (FBS, Thermo Fisher). The medium was replaced every 2 days. HFLS-RAs with a confluence above 80% at passages 4 to 10 were used in this study.

To probe into the effects of plumbagin on the HFLS-RAs, HFLS were treated with plumbagin (Sigma, USA) at different concentrations (0.125, 0.25, 0.5, 1, 1.5, 2, 2.5, 3, 3.5 μM). Since methotrexate is a folate antagonist and a first-line drug for the treatment of RA [14,15], it was used to treat HFLS-RAs at 2.2 μM as the positive control. 24, 48 and 72 hours (h) after the initiation of culture, cell viability was examined by 3-(4,5-Dimethylthiazol-2-yl)-2,5-diphenyltetrazolium bromide (MTT) assay.

Additionally, to explore the effect of plumbagin on the IL-1β-induced HFLS-RAs, IL-1β (10 ng/mL) was used to establish an inflammatory model in these HFLS-RAs [16], HFLS-RAs were treated with 10 ng/mL IL-1β for 24 h, and then treated with plumbagin (0.125, 0.25, 0.5 μM) for 48 h and then the cells were collected for following experiment.

### MTT assay

HFLS-RAs were incubated in a 96-well plate at a density of 1 × 10^4^ cells/well and cultured for 48 h (cell fusion reached 80%). After HFLSs were treated with IL-1β or plumbagin (0.125, 0.25, 0.5 μM) for 48 h, 10 µL MTT solution was added to each well as per the instructions provided by the kit (Sigma, USA) and cells were further incubated at 37°C for 4 h. The cells were subsequently centrifuged at 1000 × g for 10 minutes (min), and 100 µL DMSO was added to each well, followed by a shaking for 2 min. The optical density (OD) was detected at 450 nm, and the inhibition rate or cell viability was calculated as appropriate. This experiment was performed in independent triplicate.

### Enzyme-linked immunosorbent assay (ELISA)

The method of ELISA was used to detect the levels of TNF-α (human, ab181421; mouse, ab208348), IL-6 (human, ab178013), IL-1β (human, ab214025; mouse, ab197742), IL-17 (human, ab216167; mouse, ab199081) and RANKL (human, ab213841; mouse, ab100749). The All the commercial detection kits used were purchased from Abcam (San Francisco, California, USA), and tThe concentration was measured and calculated in line with the manufacturer’s instructions. Likewise, these experiments were conducted independently in triplicate.

### Flow cytometry

In the beginning of this assay, the splenocytes were stimulated using phorbol myristate acetate, ionomycin (Sigma-Aldrich) and GolgiStop (BD Biosciences) for 4 h. After that, the surface of cells was labeled with fluorescein isothiocyanate (FITC)-conjugated CD4 monoclonal antibodies (mAb) (eBioscience). After being permeabilized with Cytofix/Cytoperm solution, the cells were intracellularly stained with phycoerythrin (PE)-Cyanine 5 (Cy 5)-conjugated forkhead box protein 3 (Foxp3) or allophycocyanin (APC)-conjugated IL-17 (R&D Systems, Minneapolis, MN, USA). The data were finally analyzed by Accuri C6 software (BD Biosciences).

### Western blot

This assay was repeated in independent triplicate. Specifically, after HFLS-RAs treated with IL-1β and plumbagin for 48 h, HFLS-RAs were collected, and synovial tissues of mice were also collected and lysed with radio-immunoprecipitation assay (RIPA) lysis buffer. Pierce™ BCA Protein Assay Kit (23250, Thermo Fisher) was then used to determine the total protein concentration of each sample, from which 30 μg total protein was loaded, separated on the sodium dodecyl sulfate (SDS)-polyacrylamide gel at 100 V for 120 min and transferred to polyvinylidene fluoride (PVDF) membranes in sequence. After that, the membranes were blocked with 5% nonfat milk for 1 h and incubated with the following primary antibodies against MMP-1 (rabbit, 54kD, ab137332, Abcam), MMP-3 (rabbit, 54kD, ab53015, Abcam), MMP-13 (rabbit, 54kD, ab39012, Abcam), IκB (rabbit, ab32518, 36kD, Abcam), C-p65 (rabbit, #8242, 65kD, Cell signaling technology), N-p65 (rabbit, #8242, 65kD, Cell signaling technology), GAPDH (mouse, 36kD, ab8245, Abcam), and histone H2 (rabbit, #2595, 15kD, Cell signaling technology) at 4°C overnight. The membranes were subsequently washed with tris-buffered saline tween (TBST, 28360, Thermo Fisher, Waltham, Massachusetts, USA) and further incubated with the secondary antibody IgG H&L (HRP) (ab6721, Abcam, dilution ratio: 1:2000) at room temperature for 1 h. GAPDH or histone H2 was used as the internal control. For the visualization process, the membrane was developed using Pierce™ ECL plus Western blotting substrate (Thermo Fisher) in ChemiDoc MP (Bio-Rad, Hercules, California, USA). The gray value in each band was finally analyzed by Image J software (version 1.52s, National Institutes of Health, Bethesda, USA).

### Collagen-induced arthritis (CIA) animal model

Male DBA/1 mice (8 weeks, n = 45) were purchased from IMET Research Inc. (Suzhou, China). All experiments in this study were approved by the Animal Care and Use Committee of The First People’s Hospital of Yongkang.

All mice were randomly divided into 3 groups (n = 15 for each group). Namely, control group, CIA group and plumbagin (PL) group. The mice in the CIA group and the PL group were modeled using the solution of bovine type II collagen. In detail, 1.5 mL bovine type II collagen (Chondrex, USA) was mixed with an equal volume of complete Freund’s adjuvant (Sigma, USA), 0.2 mL of which was then subcutaneously injected into the tail of mouse at 1.5–2.5 cm below the base. The procedure above was repeated on day 21 using incomplete Freund’s adjuvant (Sigma, USA). Meanwhile, those in the control group did not receive treatment. In the PL group, after the first injection, plumbagin (10 mg/kg) was administered to these mice by gavage every other day from day 10 to day 50.

The clinical symptoms and score of limbs of mice in each group were observed in an independent manner by two operators blinded to the allocation of animals, and the clinical arthritis scores for each limb were assessed with a range between 0 and 3 as previously described [17]. Mice were euthanized with pentobarbital (90 mg/kg, ip) on day 50 after the first post-immunization.

### Hematoxylin-eosin (HE) staining

HE staining was employed to detect the lesions in the joint tissues of mice. In detail, the joint tissues were fixed with 4% formaldehyde and then sliced into sections with the thickness of 5 µm as needed. The prepared sections were then stained with HE staining kit (Huamei, China) for the histological observations. After the sections were sealed, the pathological state of ankle joint tissues was observed under a light microscope, and the arthritis scores were evaluated at the same time.

## Statistical analysis

The data were demonstrated as mean ± standard deviation (SD). The differences between two groups or among multiple groups were analyzed by Student’s *t*-test and one-way ANOVA. All the analyses were implemented in GraphPad 7.0 (GraphPad software, La Jolla, California, USA). *P* < 0.05 was considered to be statistically significant.

## Results

This paper mainly analyzed the effects of plumbagin on IL-1β-induced HFLS-RAs and RA-modeled mice, and unveiled its mechanism. In this study, the effects of plumbagin on the viability, inflammatory cytokines, MMPs and nuclear factor kappa-B (NF-κB) pathway of IL-1β-induced HFLS-RAs and RA-modeled mice were determined, with the evaluation on the clinical scores and histopathological changes of ankle joint of RA-modeled mice. Here, we found that plumbagin could down-regulate the levels of inflammatory cytokines and MMPs by inhibiting the activation of the NF-κB pathway, thereby attenuating RA-induced damage to HFLS-RAs and joints.

## Plumbagin inhibited the growth of HFLS-RAs

HFLS-RAs were treated with various concentrations of plumbagin, and the result showed that plumbagin exerted no significant inhibitory effect on cell viability at the concentrations of 0.125, 0.25 and 0.5 μM Figure 1(a–c). However, it should be noted that plumbagin, when given at the concentrations of 1, 1.5, 2, 2.5, 3 and 3.5 μM, inhibited the cell viability at 24, 48 and 72 h Figure 1(a–c). Meanwhile, it was found that the inhibition of cell viability induced by 1 μM plumbagin was similar to methotrexate, the drug used as the positive control Figure 1(a–c). Therefore, plumbagin was used to treat HFLS-RAs at the concentrations of 0.125, 0.25, and 0.5 μM for subsequent experiments.

**Figure 1.** Plumbagin inhibited the growth of human rheumatoid arthritis fibroblast-like synoviocytes (HFLS-RA). (a) The viability of HFLS-RA treated with different concentrations (0.125, 0.25, 0.5, 1, 1.5, 2, 2.5, 3, 3.5 μM) of plumbagin was determined by MTT assay at 24 h. The group of drug HFLS-RA treated with methotrexate was used as positive control. (b) The viability of HFLS-RA treated with different concentrations of plumbagin was determined by MTT assay at 48 h. (c) MTT assay was used to detect the effects of different concentrations of plumbagin on the growth of HFLS-RA at 72 h. *P < 0.05, **P < 0.01 vs. control group. Met: methotrexate.

## Plumbagin inhibited the levels of inflammatory factors and MMPs in HFLS under the intervention of IL-1β

To probe into the effects of plumbagin on HFLS-RAs, both plumbagin and IL-1β were used to treat these cells as appropriate. It was observable that IL-1β slightly increased the viability of HFLS-RAs, while 0.5 μM plumbagin led to a suppression on cell viability Figure 2(a).

**Figure 2.** Plumbagin inhibited the levels of inflammatory factors and matrix metalloproteinase (MMPs) of interleukin-1β (IL-1β)-treated HFLS-RAs. (a) The MTT assay was used to examine the effects of different concentrations (0.125, 0.25, 0.5 μM) of plumbagin on the viability in IL-1β (10 ng/mL)-treated HFLS-RA. (b) ELISA was used to examine the effects of different concentrations of plumbagin (0.125, 0.25, 0.5 μM) on IL-17 and RANKL levels in the IL-1β-treated HFLS-RAs. (c) ELISA was used to examine the effects of different concentrations of plumbagin (0.125, 0.25, 0.5 μM) on TNF-α and IL-6 levels in the presence of IL-1β. (d) Western blot was applied to test the effects of different concentrations of plumbagin (0.125, 0.25, 0.5 μM) on MMP-1, MMP-3 and MMP-13 protein levels. GAPDH was used as the internal control. (e) The protein expressions of MMP-1, MMP-3 and MMP-13 were quantified. ^^^^*P* < 0.01 vs. Blank; *P < 0.05, **P < 0.01 vs. IL-1β. IL-1β, interleukin-1β; TNF-α, tumor necrosis factor-α; IL-6, interleukin-6; MMP, matrix metalloproteinase.

To further analyze the mechanism through which plumbagin regulated inflammatory factors and MMPs, we divided the HFLS into five groups, namely, blank, IL-1β (10 ng/ml), IL-1β +plumbagin (0.125 μM), IL-1β + plumbagin (0.25 μM) and IL-1β + plumbagin (0.5 μM) groups. Based on the results of ELISA, IL-1β induced the release of massive inflammatory factors IL-17, RANKL, TNF-α and IL-6 in the HFLS-RAs, whereas plumbagin inhibited the secretion of IL-17, RANKL, TNF-α and IL-6 in a dose-dependent manner Figure 2(b,c). In addition, when it comes to the levels of MMPs, plumbagin dose-dependently inhibited the expression levels of MMP1, MMP3 and MMP13 proteins in HFLS-RAs in the presence of IL-1β Figure 2(d,e).

## Plumbagin regulated NF-κB pathway

Additionally, we investigated the effects of plumbagin on NF-κB pathway in HFLS-RAs, and the results demonstrated that IL-1β remarkably inhibited the levels of IκB and cytoplasmic p65 (C-p65), while promoting the protein level of nuclear p65 (N-p65). On the contrary, plumbagin at the concentration of 0.5 μM could significantly up-regulate the levels of IκB and C-p65 yet down-regulate that of N-p65 in HFLS with the presence of IL-1β Figure 3(a–c).

**Figure 3.** Plumbagin could regulate NF-κB pathway. (a) Western blot was applied to detect the protein expression of IκB, C-p65 and N-p65 after HFLS-RA were treated with 10 ng/mL IL-1β and 0.5 μM plumbagin. GAPDH or histone H2 was used as the internal control. (b) The protein expressions of IκB and C-p65 were quantified. (c) The protein expression of N-p65 was quantified. ^&&^*P* < 0.01 vs. Blank; *P < 0.05, **P < 0.01 vs. IL-1β; ^^^^*P* < 0.01 vs. 0.5 μM plumbagin. C-p65, cytoplasm p65; N-p65, nucleus p65; IL-1β, interleukin-1β.

## Plumbagin could alleviate the symptoms of RA in CIA mice, inhibit inflammatory factors and MMPs, and regulate NF-κB pathway

Likewise, the RA model was established in mice with CIA as the inducer, and the mice were treated with plumbagin as well. The results of HE staining verified that compared with the mice in the control group, inflammatory cell infiltration, cartilage destruction, joint stenosis, and synovial hyperplasia were observed in the ankle joint tissues of mice of the OA group Figure 4(a). Such inflammatory cell infiltration and cartilage destruction were markedly reduced in mice of the PL group compared to those in the OA group Figure 4(a). Meanwhile, the clinical scores of the PL group mice were also greatly lower than those of the OA group mice Figure 4(b).

**Figure 4.** Plumbagin could alleviate rheumatoid arthritis (RA) in collagen-induced arthritis (CIA) mice, inhibit inflammatory factors and MMPs, and regulate NF-κB pathway. (a) HE staining was used to detect the ankle joint tissue of CIA mice. (b) Joint clinical scores were used to analyze the effects of plumbagin on joint damage in CIA mice. (c) Representative flow cytometry profile and quantification (d) of IL-17+ and Foxp3+ cells in splenic CD4 + T cells isolated from CIA mice. (e-f) ELISA was used to detect the effects of plumbagin on IL-17 and RANKL in the connective tissues and serum of CIA mice. (g) The effect of plumbagin on tumor necrosis factor-α (TNF-α) and interleukin-1β (IL-1β) in connective tissues of CIA mice. (h) ELISA was used to detect the effects of plumbagin on TNF-α and IL-1β in the serum of CIA mice. (i) Western blot was applied to test the effects of plumbagin on matrix metalloproteinase (MMP)-1, MMP-3, and MMP-13 protein. GAPDH was used as the internal control. (j) The protein expressions of MMP-1, MMP-3 and MMP-13 were quantified. (k) Western blot was applied to test the effects of plumbagin on the IκB and N-p65 protein. GAPDH or histone H2 was used as the internal control. (l) The protein expressions of IκB and N-p65 were quantified. ^^^^*P* < 0.01 vs. Control; *P < 0.05, **P < 0.01 vs. CIA group. PL, plumbagin; N-p65, nucleus p65. 10 mg/kg plumbagin was used in in vivo experiment.

As for the inflammatory factors, in contrast with those in the OA group, in mice of the PL group, the level of Foxp3 was increased Figure 4(c,d), while the levels of IL-17 and RANKL were lower Figure 4(e,f). Additionally, the levels of TNF-α, IL-6, MMP1, MMP3 and MMP13 in the OA group were dramatically promoted, while the above-mentioned factors levels in the PL group were significantly lower than those in the OA group Figure 4(g–j).

Finally, the levels of NF-κB pathway-related factors were detected, where we confirmed that as compared those allocated to the OA group, the protein level of IκB was noticeably higher yet the level of N-p65 protein was evidently lower in the PL group Figure 4(k,l).

## Discussion

In the pathogenesis of RA, fibroblast-like synoviocytes (FLS) are the ultimate effector cells of RA-induced joint injury. FLS stimulates or inhibits inflammatory response under autocrine or paracrine modes through regulating the expression signals such as cytokines and chemokines [18]. Considering synovial cell proliferation and cytokine oversecretion are the main mechanisms of RA, we first analyzed the effects of plumbagin on HFLS-RAs, with methotrexate as the positive control [19]. It was confirmed in the results of this study that compared with the cells treated with high concentration of plumbagin, the inhibitory effect of plumbagin on cell viability was weaker at the concentration of 0.125, 0.25 and 0.5 μM. Moreover, the inhibition of cell viability induced by plumbagin at the concentration of 1 μM was similar to the positive control drug methotrexate, in addition to the discovery that plumbagin exerted a strong inhibitory effect on the cell viability at the concentration of 1.5, 2, 2.5, 3 and 3.5 μM. It was thus suggested that plumbagin has an inhibitory effect on the proliferation of FLS, and this chemical at the concentrations of 0.125, 0.25 and 0.5 μM were used in subsequent experiments.

IL-1β has been documented as a pivotal pathogenic mediator during RA [20,21]. Oversecretion of IL-1β can stimulate synovial and chondrocyte synthesis, and release prostaglandin E2, collagenase and inflammatory factors, triggering synovial inflammation and cartilage matrix disintegrates [22,23]. Meanwhile, IL-1β promotes the aggregation of neutrophils, lymphocytes and macrophages by acting on endothelial cells, and aggravates the local inflammatory response of joints [22,23]. The effect and target cells of TNF-α are similar to IL-1β, and the secretion of TNF-α can also promote the synthesis and secretion of IL-1β, which is a positive feedback regulation [24,25]. In this study, we discovered that IL-1β promoted the secretion of TNF-α and IL-6 from HFLS-RAs, while plumbagin did the opposite, indicating that plumbagin treatment could alleviate the RA-induced inflammatory response. MMPs can almost hydrolyze various protein components of the extracellular matrix, leading to the destruction of joint ligaments, bones and cartilage [26]. MMP-3 is an important protease for the induction of cartilage degradation, which can act as an indicator of synovial damage and prognosis of patients with RA [27]. MMP-1 and MMP-13 are also important participants in RA cartilage injury [26,28]. It has been reported that miR-4423-3p inhibits the proliferation of HFLS-RAs by targeting MMP-13 [29]. Here, owing to the notable inhibitory effects on the expressions of MMP-1, MMP-3 and MMP-13 in IL-1β-induced HFLS-RAs, the treatment of plumbagin was proved to significantly attenuate the RA-induced tissue damage. Existing studies have proposed that plumbagin can suppress the epithelial-mesenchymal transition of retinal pigment epithelial cells by inhibiting the level of MMPs *in vivo* and *in vitro* [30]. Zhang et al. [31] further demonstrated that plumbagin can attenuate the inflammation by regulating pyruvate kinase M2 (PKM2). Likewise, in the study, it becomes clear that plumbagin could inhibit the excessive secretion of TNF-α, IL-6 and MMPs in HFLS-RAs induced by IL-1β so as to suppress RA-related inflammation and tissue injuries.

To further analyze the mechanism of plumbagin, we examined the effect of plumbagin on CIA mice, the results of which indicated that plumbagin remarkably inhibited joint damage in CIA mice, and suppressed the levels of inflammatory cytokines and MMPs in their joint tissues. Following the activation of NF-κB pathway, one of the vital pathways of inflammatory response, p65 will transfer from the cytoplasm into the nucleus, bind to corresponding inflammation-related genes, and initiate transcription of inflammatory cytokines, thereby inducing inflammation [32,33]. As an inhibitor of NF-κB, IκB inhibits the activation of the NF-κB pathway [34] that can promote the expression of MMPs [35,36]. Additionally, it’s worth noting that plumbagin could also significantly up-regulate the levels of IκB and p65 in the cytoplasm, and inhibit the activation of NF-κB. Studies have proved that the activation of NF-κB acts as an important mechanism in RA [37,38]. For example, β-arrestin-2 alleviates RA-associated injury by suppressing the activation of NLRP3 inflammasome and NF-κB pathway in macrophages [39]. As for plumbagin, it could inactivate NF-κB and alleviate the inflammatory response of H_2_O_2_-induced neurons [40,41]. Zaki et al. [42] has additionally pointed out that plumbagin can inhibit the NF-κB pathway by modulating high mobility group box 1, confirming the possible effect of plumbagin on RA. In our current investigation, plumbagin could down-regulate the expressions of inflammatory factors and MMPs by up-regulating IκB and inhibiting the activation of NF-κB so as to reduce joint damage caused by RA.

In addition, regulating the immune response plays an important role in the improvement of RA. Plumbagin inhibits the mitogen-induced T-cell proliferation and cytokine (IL-2/IL-4/IL-6/IFN-γ) production of lymphocytes [43]. It has been reported that the reduced IgG2a responses by plumbagin could influence the anti-inflammatory cytokine secretion by stimulating Th1 cells in CIA mice [44]. Meanwhile, plumbagin is proved useful for treating bone-related diseases, and exerts its biological activities primarily through inducing reactive oxygen species and triggering osteoblast-mediated bone formation [45]. These studies indicated that plumbagin is indeed effective in the mechanism based treatment of RA, suggesting that plumbagin may be used as an alternative treatment to methotrexate in RA. However, some limitations of this study should be noted. For instance, the use of NF-κB pathway agonists should be included to further verify the role of plumbagin and its interaction with NF-κB pathway in RA. Meanwhile, further research is needed on the efficacy and mechanism of plumbagin in RA. For instance, it remains vague whether plumbagin can regulate the roles of other pathways or specific target genes in RA. Furthermore, in order to further evaluate the efficacy of plumbagin, a comparison should be made in plumbagin and those approved RA therapies concerning the therapeutic potential.

## Conclusion

In this study, plumbagin could inhibit the levels of inflammatory cytokines and MMPs by inhibiting the activation of the NF-κB pathway, thereby attenuating RA-induced damage to cells and joints. Plumbagin treatment reduced the inflammatory response of RA and joint tissue damage, proving that plumbagin may be an effective therapeutic drug for RA, which sheds new light on the clinical treatment of RA and enriches the knowledge of using traditional Chinese medicine in the treatment of arthritis.

## Supplementary Material

Supplemental Material

## Data Availability

The analyzed data sets generated during the study are available from the corresponding author on reasonable request.
